The article "Analysis of Related Factors of Early Mortality in Patients with Severe Renal Injury Treated with Continuous Venovenous Hemodialysis" was published in 2022. Journal: J Healthc Eng.

# Analysis of Related Factors of Early Mortality in Patients with Severe Renal Injury Treated with Continuous Venovenous Hemodialysis

**DOI:** 10.1155/2022/7812788

**Published:** 2022-01-25

**Authors:** Qingyun Wang, Jia Liu, Chengquan Zhai, Juan Liu

**Affiliations:** ^1^Blood Purification Room, Jinan Municipal Hospital of Traditional Chinese Medicine, Jinan City 250012, Shandong Province, China; ^2^Department of Critical Care Medicine, Yantai Yuhuangding Hospital, Yantai 264000, Shandong Province, China; ^3^Department of Emergency, Zaozhuang Municipal Hospital, Zaozhuang City 277100, Shandong Province, China; ^4^Department of Hemodialysis, Beijing Fengtai Hospital of Integrated Traditional Chinese and Western Medicine, Beijing 100072, China

## Abstract

**Background:**

To explore the related factors of early mortality in patients with severe renal injury treated with continuous venovenous hemodialysis (CVVHD), this study is of great significance to improve the treatment effect of hemodialysis.

**Methods:**

Clinical data of 83 patients with severe renal injury who underwent CVVHD treatment in Nephrology Department of our hospital (January 1, 2017, to June 30, 2019) were retrospectively analyzed.

**Results:**

Mortality was the highest in the first month of CVVHD treatment and then decreased obviously. Early mortality was particularly higher in patients aged 60 and above. Age of first hemodialysis, cardio cerebrovascular diseases, serum phosphorus, urea nitrogen, blood calcium, platelet count, lean body mass (LBM), and total cholesterol were significant risk factors for early mortality.

**Conclusion:**

The early mortality of patients with severe renal injury during CVVHD treatment was higher.

## 1. Introduction 

Severe renal injury refers to a rapid decline in renal function caused by a variety of factors. The latest data survey shows that there were 1.4 million and 2.9 million hospitalized patients with severe renal injury in China in 2018, with a total medical cost of 13 billion US dollars [1, 2]. The in-hospital mortality rate of patients was 12.4%, and about 65.3% of patients died within 3 months after discharge [3]. Continuous venovenous hemodialysis (CVVHD) is a common treatment for renal diseases, which can slowly and continuously remove the excess water and toxic substances from the patients with the main effect of convection and adsorption, and is more conducive to clearing large and medium molecules such as cytokines and immune complexes. With the development of hemodialysis treatment technology, the survival of patients treated with hemodialysis has been improved, but some patients still die from complications such as cerebral edema, renal hypertension, and renal osteodystrophy [4–6]. The definition of early death is that patients die within 90 days after first CVVHD treatment [7, 8]. Previous studies have found that cardiovascular diseases, age, and blood calcium levels are risk factors of mortality in patients with renal injury, and temporary conduit for first vascular access and complicated tumor will also increase the early mortality risk of patients to some extent [7]. However, Carolyn et al. found that total cholesterol and diabetes are also risk factors of death [9]. However, there are no studies pointing out the relevant factors affecting early death of patients undergoing CVVHD. Therefore, to explore the related risk factors of early mortality in dialysis patients and provide more evident-based basis for reducing the early dialysis mortality, clinical data of 83 patients with severe renal injury who underwent CVVHD treatment in Nephrology Department of our hospital (January 1, 2017, to June 30, 2019) were retrospectively analyzed, so as to reduce the early mortality and improve the treatment effect.

## 2. Materials and Methods

### 2.1. General Data

Clinical data of 83 patients with severe renal injury who underwent CVVHD treatment in Nephrology Department of our hospital (January 1, 2017 to June 30, 2019) were retrospectively analyzed. Patients were followed up until June 30, 2020.

### 2.2. Inclusion and Exclusion Criteria

#### 2.2.1. Inclusion Criteria

(1) Patients met the diagnostic criteria in KDIGO Clinical Practice Guideline for Acute Kidney Injury [10], with the clinical manifestations including eyelid or bilateral lower extremity edema, oliguria, elevated blood pressure, and nausea and vomiting. (2) Patients received regular hemodialysis treatment, to be specific, weekly dialysis time ≥12 hours, more than 4 hours each time and 3 times per week, or more than 6 hours each time and 2 times a week. (3) The study met the World Medical Association Declaration of Helsinki (2013) [11].

#### 2.2.2. Exclusion Criteria

(1) Patients were registered repeatedly. (2) Clinical data of patients were missing. (3) Patients were under the age of 18. (4) Patients were treated with peritoneal dialysis or renal transplantation before CVVHD treatment.

#### 2.2.3. Methods

Patients' clinical data of age, gender, age of first hemodialysis, and basic diseases were recorded. 5 ml of fasting cubital venous blood was collected from the patients to measure related indexes, including serum phosphorus, serum albumin, blood calcium, urea nitrogen, platelet count, total cholesterol, triacylglycerol, C-reactive protein, hemoglobin, blood magnesium, and serum creatinine. Meanwhile, lean body mass (LBM) of patients was calculated. LBM = 0.34 × serum creatinine (mg/dl, 1 mg/d1 = 88.4 *μ*mol/L) + 5.58 × gender (1 for women and 0 for men) + 0.30 × body mass (kg) + 0.67 × height (inch) − 0.23 × urea clearance rate − 5.75 (inch = 0.1254 m) [12].

The mortality within 6 months of hemodialysis treatment was recorded. Mortality = number of deaths within the time period/number of exposures within the time period. See Figure 1 for specific flow chart of the research.

### 2.3. Statistical Methods

All experimental data of the study were processed by SPSS23.0, and the pictures were graphed by GraphPad Prism 7 (GraphPad Software, San Diego, USA). Enumeration data were tested by *x*^2^ and expressed by [*n* (%)]. Measurement data were tested by *t* expressed by mean ± SD. The Cox regression model was used to analyze the risk factors of early mortality in patients treated with hemodialysis. The differences were statistically significant at *P* < 0.05.

## 3. Results

### 3.1. General Data of Patients

See Table 1 for details.

### 3.2. Analysis of Laboratory Indexes of Patients

See Table 2 for details.

### 3.3. Comparison of Mortality at Different Time Points within 6 Months of Hemodialysis Treatment

The mortality of patients within 6 months of hemodialysis treatment was statistically analyzed, which was highest within the first month, and then decreased significantly (see Figure 2).

### 3.4. Correlation between LBM and Early Mortality

After follow-up, according to different LBM values (<36.7, 36.7–40.5, 40.6–44.9, 45.0–49.4, and >49.4), patients were divided into five groups, and the crude mortality of the 5 groups was 35.29%, 31.25%, 26.67%, 17.65%, and 11.11%, respectively (see Table 3).

### 3.5. Analysis of Related Factors of Early Mortality

Age, cardiovascular disease, blood phosphorus, blood calcium, platelet count, LBM value, total cholesterol, and urea nitrogen are independent risk factors of early mortality in patients treated with hemodialysis (see Table 4).

### 3.6. Correlation Analysis of Early Mortality of Patients Treated with Hemodialysis

See Figure 3 for details.

### 3.7. Comparison of Area of Each Single Index Item, Standard Error, Asymptotic Significance, and Asymptotic 95% Confidence Interval

The age of first hemodialysis was higher than that of other single tests (see Table 5).

### 3.8. Comparison of Positive Cases and Sensitivity of Each Index

Sensitivity of age of first hemodialysis was the highest (see Table 6).

## 4. Discussion

Continuous hemodialysis is a common method for the treatment of severe renal injury at present, which is the improvement of intermittent dialysis treatment technology. Through slow flow rate of dialysis fluid and the principle of convection and dispersion [13, 14], this treatment method can realize blood highly purification by removing water molecules and solute exchange. With more displacement liquid and longer dialysis duration [15], toxic components in patients' blood can be effectively removed, which can achieve ideal treatment effect, and its efficacy has been confirmed in diseases such as diabetic ketoacidosis and multiple organ dysfunction syndrome [16]. However, clinical research shows that some patients die within 90 days of hemodialysis treatment [17], so it is important to actively explore and prevent the related factors of early mortality in patients with severe renal injury treated with hemodialysis.

Through retrospective analysis, this study found that the highest overall mortality rate of patients was observed in the first month of hemodialysis treatment, reaching 51.36%, which was similar to the conclusion of a foreign study [18]. The foreign study confirmed that the mortality rate in the first month of hemodialysis was the highest, with 41.28%, 43.28%, and 45.19% in Germany, Britain, and Canada, respectively, within 30 days, which may be related to comorbidities, primary diseases, health policies, and cultures of patients in different countries. Cox regression model analysis found that the age of the first hemodialysis was closely related to the early mortality which was particularly higher in patients aged 60 and above. It is speculated that this is due to the complicated complications of elderly patients and decreased willpower and cognitive function, so the quality of life is usually affected and the mortality increases during hemodialysis treatment [19–21]. Platelet factors play an important role in the smooth progress of dialysis, and studies have confirmed that an increased number of platelets can increase the patients' blood viscosity, which can lead to thrombosis and increase the risk of death. Abnormalities in serum calcium can lead to disorders in calcium phosphate metabolism and accelerate the progression of vascular calcification, thereby greatly increasing the occurrence of cardiovascular disease and, to a greater extent, the risk of death in dialysis patients. In addition, the increase in urea nitrogen in patients indicates a serious decline in renal function [22], which leads to a relatively serious condition and even an increase in early mortality. Another study found that the incidence of protein energy consumption (PEW) and reflex sympathetic dystrophy syndrome (RSDS) in patients treated with hemodialysis was higher [23]. Compared with the healthy people, LBM values in hemodialysis patients significantly decreased. Some scholars believe that PEW is an independent and significant factor to predict the death of hemodialysis patients [24], so a higher LBM value represents a better nutritional level and reflects a higher survival rate of patients. This study found that the mortality rate of the group (LBM > 49.4) was 11.11%, which is lower than that of the other groups.

There are some defects in this study. First, all the cases selected in this study were patients from local hospitals, so the source of cases was single. Second, the study only included some relevant indexes before hemodialysis, without the analysis of clinical data during hemodialysis treatment. Finally, the study included a small sample size and lacked comprehensiveness, so the conclusions obtained in this study remain to be improved by further studies.

To sum up, the early mortality of patients with severe renal injury during CVVHD treatment was higher. Age of first hemodialysis, comorbid cardio cerebrovascular diseases, serum phosphorus, urea nitrogen, blood calcium, platelet count, lean body mass (LBM), and total cholesterol were significant risk factors for early mortality. Therefore, the above risk factors should be actively prevented to improve clinical prognosis.

## Figures and Tables

**Figure 1:** Research process.

**Figure 2:** Mortality at different time points within 6 months of hemodialysis treatment. *Note*. The abscissa indicates months and the ordinate indicates mortality (%).

**Figure 3:** Correlation analysis of early mortality of patients treated with hemodialysis.

**Table 1:** General data of patients [*n* (%)].

Item	Number of cases	Percentage (%)
Gender		
Male	47	56.63
Female	36	43.37

Age		
18–26 years old	16	19.28
27–46 years old	29	34.94
47–60 years old	25	30.12
Over 60 years old	13	15.66

Basic diseases		
Hypertension	61	73.49
Diabetes	35	42.17
Hyperuricemia	19	22.89
Hypotension	13	30.12

Residence		
Urban	35	42.17
Rural	48	57.83

Educational degree		
University degree	14	16.87
Middle school	53	63.86
Primary school	16	19.28

**Table 2:** Analysis of laboratory indexes of patients (mean ± SD).

Item	Value
Serum phosphorus (mmol/L)	1.74 ± 0.48
Serum albumin (g/L)	34.19 ± 5.87
Blood calcium (mmol/L)	2.41 ± 0.41
Urea nitrogen (mmol/L)	15.67 ± 2.36
Platelet count (10^9^/L)	281 ± 83.27
Total cholesterol (mmol/L)	9.24 ± 1.35
Triacylglycerols (mmol/L)	1.42 ± 0.36
C-reactive protein (mg/L)	47.24 ± 0.45
Hemoglobin (g/L)	85.48 ± 13.28
Blood magnesium (mmol/L)	0.42 ± 0.14
Serum creatinine (*μ*mol/L)	131.22 ± 18.35

**Table 3:** Comparison of survival rate of 83 patients treated by CVVHD and grouped according to LBM values [*n* (%), mean ± SD].

Group	*n*	Crude mortality	Uncorrected model		Case correction model		Case correction and MICS model	
			*P*	HR (95% CI)	*P*	HR (95% CI)	*P*	HR (95% CI)
<36.7	17	6 (35.29%)	0.021^a^	1.32 (1.02, 1.56)	0.039^a^	1.49 (1.32, 1.67)	0.041^a^	1.32 (1.07, 1.48)
36.7–40.5	16	5 (31.25%)	0.058	1.06 (0.96, 1.35)	0.064	1.24 (1.05, 1.32)	0.054	1.19 (1.06, 1.43)
40.6–44.9	15	4 (26.67%)						
45.0–49.4	17	3 (17.65%)	0.052	0.96 (0.68, 1.15)	0.059	0.92 (0.73, 1.24)	0.052	0.82 (0.72, 0.93)
>49.4	18	2 (11.11%)	0.057	0.92 (0.73, 1.25)	0.036^a^	0.75 (0.63, 0.89)	0.035^a^	0.83 (0.74, 0.96)

*Note.* ‘a' indicates *P* < 0.05.

**Table 4:** Analysis of related factors of early mortality.

Item	HR	95% CI	*P*
Age (≥60 years old)	1.865	1.253–2.845	<0.001
Gender (male)	1.024	0.683–1.473	0.746
Complicated with cardiovascular disease	1.572	0.732–2.414	0.041
Serum phosphorus (mmol/L)	1.437	0.836–2.364	0.013
Blood calcium (mmol/L)	1.527	0.735–2.176	0.023
Platelet count (10^9^/L)	1.367	0.826–2.073	0.031
Lean body mass (LBM) (kg)	1.462	0.738–1.957	0.024
Total cholesterol (mmol/L)	1.637	0.983–2.167	0.034
C-reactive protein (mg/L)	1.243	0.625–1.834	0.856
Triacylglycerols (mmol/L)	1.352	0.753–1.736	0.753
Serum albumin (g/L)	1.263	0.746–1.538	0.653
Urea nitrogen (mmol/L)	0.945	0.537–1.254	0.036
Hemoglobin (g/L)	1.036	0.638–1.574	0.326
Blood magnesium (mmol/L)	0.835	0.537–1.352	0.825
Serum creatinine (*μ*mol/L)	1.162	0.627–1.568	0.479

**Table 5:** Area under curve.

Test result variables	Area	Standard error	Asymptotic significance	Asymptotic 95% confidence interval	
				Lower limit	Upper limit
Age of first hemodialysis	0.882	0.038	0.000	0.808	0.957
Cardiovascular and cerebrovascular diseases	0.833	0.044	0.000	0.747	0.920
Blood phosphorus	0.784	0.049	0.000	0.688	0.881
Urea nitrogen	0.804	0.047	0.000	0.711	0.897
Blood calcium	0.775	0.050	0.000	0.676	0.873
Platelet count	0.804	0.047	0.000	0.711	0.897
Lean body mass (LBM)	0.745	0.053	0.000	0.642	0.848
Total cholesterol	0.775	0.050	0.000	0.676	0.873

**Table 6:** Diagnostic results of each index.

Index	Age of first hemodialysis	Cardiovascular and cerebrovascular diseases	Blood phosphorus	Urea nitrogen	Blood calcium	Platelet count	Lean body mass (LBM)	Total cholesterol
Positive (cases)	39	34	29	31	28	31	25	28
Sensitivity	80.95	75.00	69.86	71.83	68.92	71.83	66.23	68.92

## Data Availability

The data used to support the findings of this study are available upon reasonable request from the corresponding author.
